The article "Preliminary validity of the BNSSS-20 in Arabic: Exploratory study on basic needs satisfaction in sport for a sample of Tunisian athletes" was retracted in 2025. Reasons: unreliable data; unreliable results or conclusions; lack of ethics approval or compliance; missing or withdrawn patient consent.

# Preliminary validity of the BNSSS-20 in Arabic: Exploratory study on basic needs satisfaction in sport for a sample of Tunisian athletes

**DOI:** 10.1371/journal.pone.0294582

**Published:** 2023-11-16

**Authors:** Mohamed Baaziz, Ali Aloui, Saber Abdellaoui, Matthew Stults-Kolehmainen, Daniel Boullosa, Abderraouf Ben Abderrahman

**Affiliations:** 1 Higher Institute of Sport and Physical Education of Ksar-Said, University of Manouba, Manouba, Tunisia; 2 Division of Digestive Health, Yale New Haven Hospital, New Haven, CT, United States of America; 3 Department of Biobehavioral Sciences, Teachers College–Columbia University, New York, NY, United States of America; 4 Catholic University of Brasilia, Taguatinga, Brazil; National Cheng Kung University College of Medicine, TAIWAN

## Abstract

**Background:**

Satisfaction of fundamental needs is an important concept in sport, but currently there is no tool in Arabic to measure this construct. Basic needs are often linked to high rates of motivation and performance. It is necessary to develop tools to assess psychological needs in the sport context.

**Aim:**

This study aimed to validate the Basic Needs Satisfaction in Sport Scale (BNSSS) in Arabic language across Tunisian athletes, and to test its psychometric properties (factorial structure, internal reliability, construct validity, and sensitivity).

**Methods:**

Athletes in various sports participated in this study (370 men, 146 women; mean age 18.35) and voluntarily completed the Arabic version of the BNSSS-20. Both exploratory (EFA, *N* = 294; males: 68%; females: 32%; [14–18] = 182; [19–28] = 112) and confirmatory (CFA; *N* = 222; males: 76.6%; females: 23.4%; [14–18] = 103; [19–28] = 119) factor analyses were examined.

**Results:**

Results from the EFA suggest that the BNSSS scale reflects the theoretical model well, with good internal consistency for all factors. All 20 items of BNSSS revealed excellent reliability (McDonald’s omega = 0.773, Cronbach’s α = 0.886, Gutmann’s λ6 = 0.970) and good temporal stability (ICC = 0.84, 95% CI = 0.55–0.93) over a 4-week period. Likewise, the CFA fit indices were excellent.

**Conclusion:**

The BNSSS presented excellent fit to the theoretical model for all indices, confirming the factorial structure and providing validity of the instrument for Tunisian athletes.

## Introduction

Self-determination theory (SDT) is centered around several sub-theories [1, 2]: cognitive appraisal theory [3], causal orientations theory [4], organismic integration theory [5], and basic needs theory [6], each addressing specific theoretical features, yet connected by the concept of basic psychological needs and an organismic and dialectic meta-theory Standage [7]. Deci and Ryan [8] suggest that the intrinsic motivated behavior is related to the satisfaction of the three basic psychological needs. Cognitive evaluation theory indicates that an intrinsically motivated individual is always seeking to satisfy three basic and universal needs (i.e., autonomy, competence, and relatedness) [3, 9]. Studies on SDT have emphasized that these needs must be fulfilled in order to maintain functional mental health [10, 11] individual well-being [2, 5, 10, 11], and personal motivation [6, 12].

The article "Preliminary validity of the BNSSS-20 in Arabic: Exploratory study on basic needs satisfaction in sport for a sample of Tunisian athletes" was retracted in 2025. Reasons: unreliable data; unreliable results or conclusions; lack of ethics approval or compliance; missing or withdrawn patient consent.

Self-determination theory in a sporting domain has been a great deal of research in recent years [13–15], indicating the importance of basic needs [13, 16]. To start, the need for competence in skill leads to the desire to interact effectively with one’s environment while performing activities that are within one’s abilities [17]. The need for competency leads individuals to match challenges to their abilities and to develop them according to their desired activities [5]. Vlachopoulos and Michailidou [18] found that the need for competency encompasses the strongest component of motivation for physical activity. Second, Reeve, Nix [19] proposed merging the autonomy-internal perceived locus of causality and autonomy-volition aspects in the education context. Ng, Lonsdale [20] initially suggested three-factor type of autonomy model because the relations between autonomy concepts may change in the sport context. First, the internal locus of perceived causality (IPLOC) refers to whether an individual believes that his or her actions are initiated and regulated by a personal force. Second, volition indicates an unpressured willingness to embark in an activity. Finally, perceived choice relates to the perception of having decision-making flexibility to choose whether to participate in an activity. Third, the need for relatedness indicates the need to be connected with other individuals in one’s social environment by highlighting the importance of interaction with these individuals [21]. The need for relatedness is the feeling of meaningful association with others [22]. This need for affiliation, however, depends on the social domain in which the person inhabits, such as sport [23, 24]. The perceived satisfaction of these needs are determined by the individual specifics of the form of motivation, that in turn drives their overall well-being and behaviors [6]. Ng, Lonsdale [20] have suggested that the fulfilment satisfaction of these needs is predictive of intrinsic motivation. These three needs have an effect on an athlete’s intrinsic motivation. Furthermore, frustration of these needs has a negative impact on anxiety [25] and depression [26]. SDT indicates that needs intervene at human development Ryan [27]. According to Ryan and Deci [28], these needs concern all individuals, irrespective of their culture, gender or age.

The article "Preliminary validity of the BNSSS-20 in Arabic: Exploratory study on basic needs satisfaction in sport for a sample of Tunisian athletes" was retracted in 2025. Reasons: unreliable data; unreliable results or conclusions; lack of ethics approval or compliance; missing or withdrawn patient consent.

Various studies have delineated the benefits of satisfying basic needs (e.g., well-being; Murcia and Sánchez-Latorre [29], work; Sánchez-Oliva, Morin [30], and education; Méndez-Giménez and Pallasá Manteca [31]). On the contrary, unfulfillment of these three basic needs causes negative consequences on health and psychological well-being or even leads to the total absence of motivation, sometimes called amotivation [32].

Several authors have made progress in producing measures of needs satisfaction in a variety of life domains, including work, exercise and sport. Gagné [33] studied the factors that influence motivation and assessed satisfaction needs by developing the Basic Psychological Needs at Work Scale (BPNWS). An adaptation was also made in the area of physical activity—Vlachopoulos and Michailidou [18] created the Basic Psychological Needs in Exercise Scale (BPNES). This instrument consists of 12 items—four items for each of three dimensions (autonomy, competency, and affiliation). The internal consistency of the scale acceptable, with good results determined a valid fit for the hypothesized model. Similarly, Wilson, Rogers [34] established the Psychological Needs Satisfaction in Exercise Scale. This tool includes 18 items—six items for each dimension (autonomy, competence, and relatedness). The internal consistency of the instrument is excellent, with good model fit indices.

Gillet, Rosnet [22] organized the psychological needs satisfaction scale. This instrument consists of 15 items—five sub-items for each dimension (competence, autonomy, and relationship). Ng, Lonsdale [20] detailed the need for autonomy by developing the Basic Needs Satisfaction in Sport Scale (BNSSS) specifically for the competitive sport domain with affiliated athletes. The BNSSS has 20 items; five items each for two dimensions (competence (COMP) and relatedness (RELAT)) while autonomy only contains 10 items. Based on expert opinion in the sport context, these authors divided autonomy into three subscales: four items for autonomy-choice (Auto.choice), three items for autonomy-volition (Auto.volition) and three items for autonomy-internal perceived locus of causality (IPLOC). Cronbach’s alpha coefficients produced good values (Auto.choice was 0.82, 0.76 for IPLOC, 0.77 for COMP, 0.61 for Auto.volition, and 0.87 for RELAT). The model fit indices confirmed good results (NNFI = 0.96; CFI = 0.97; RMSEA = 0.06; and the standardized root mean square residual (SRMR) = 0.07).

The article "Preliminary validity of the BNSSS-20 in Arabic: Exploratory study on basic needs satisfaction in sport for a sample of Tunisian athletes" was retracted in 2025. Reasons: unreliable data; unreliable results or conclusions; lack of ethics approval or compliance; missing or withdrawn patient consent.

More recently, Nascimento Junior, Nickening Vissoci [35] validated the Brazilian Version of the Basic Needs Satisfaction in Sport Scale. The tested model indices of 20 items showed the existence of three factors (autonomy, competence, and relatedness). However, the fit of this model was unsatisfactory (χ ^2^ (167) = 871.25; χ ^2^/df = 5.217; CFI = 0.73; GFI = 0.80; TLI = 0.70; RMSEA = 0.10 (0.09–0.11); (RMSEA < 0.05); *p* = 0.001). These authors proposed a new acceptable version composed of 12 items. Confirmatory factor analysis confirmed a new model with acceptable values that are close to the critical values (Adjusted goodness of fit statistic (AGFI) = 0.90; Goodness of Fit Index (GFI) = 0.93; Tucker-Lewis Index (TLI) = 0.89; RMSEA = 0.08). Pineda-Espejel, López Gaspar [36] created a Spanish version of the BNSSS adapted in Mexico. The results demonstrated good psychometric properties to measure satisfaction of the three basic needs (autonomy, competence, and relatedness) after the deletion of one item. Also, Gümüşay and Argan [37] validated a Turkish version of BNSSS that had 14 items. The CFA results provided good psychometric properties (Chi-Square/df = 1.84, RMSEA = 0.071, RMR = 0.028, SRMR = 0.057, Bentler-Bonett non normed fit index (NFI) = 0.92, NNFI = 0.95, CFI = 0.96, GFI = 0.90, and AGFI = 0.85).

Research on basic needs in sports is currently limited in Arabic-speaking countries. The work of basic needs in the sport context by insisting on each aspect of this basic needs might help coaches and researchers in Arab countries to identify effective interventions that could enhance the motivation, performance, and experiences of athletes. We will thus try to better understand the aspects that explain his needs (i.e., autonomy, competence and affiliation) among the athlete. Therefore, the purpose of this study was to adapt an Arabic version of the BNSSS and test its psychometric properties in a large sample of male and female Tunisian athletes in multiple sports. To test reliability of the translated and adapted scale, we followed a subset of athletes across four weeks.

## Methods and equipment

### Population

Our population is composed of 516 national- and international-caliber athletes (370 male athletes, 146 female athletes; mean age 18.35 ± 3.43 years; 14 to 28). This population practices various competitive disciplines: 378 athletes were in team sports (soccer, handball, volleyball, and basketball) and 138 athletes were in individual sports (kick boxing, English boxing, Taekwondo, athletics, gymnastics, and swimming). Table 1 contains general information about the study sample (mean, standard deviation, skewness, and kurtosis). 516 responses (males: 71.7%; females: 28.3%) of the 530 responses were retained for the final analysis; 14 were excluded for missing responses. The geographical distribution of the participants was as follows: Tunis (22.1%), Sfax (19.8%), Kairouan (19.6%), Gafsa (21.3%), and Gabes (17.2%).

The article "Preliminary validity of the BNSSS-20 in Arabic: Exploratory study on basic needs satisfaction in sport for a sample of Tunisian athletes" was retracted in 2025. Reasons: unreliable data; unreliable results or conclusions; lack of ethics approval or compliance; missing or withdrawn patient consent.

**Table 1:** Basic characteristics of the sample population.

Variable		Effective			Pourcentage (%)
Age		[14–18]	Total (*N* = 516)	313	60.70
			EFA (*n* = 294)	182	61.90
			CFA (*n* = 222)	103	46.40
			Test-retest (*n* = 37)	14	37.80
		[19–28]	Total (*N* = 516)	203	39.30
			EFA (*n* = 294)	112	38.10
			CFA (*n* = 222)	119	53.60
			Test-retest (*n* = 37)	23	83.80
Gender		Male	Total (*N* = 516)	370	71.70
			EFA (*n* = 294)	200	68
			CFA (*n* = 222)	170	76.60
			Test-retest (*n* = 37)	16	43.20
		Female	Total (*N* = 516)	146	28.30
			EFA (*n* = 294)	94	32
			CFA (*n* = 222)	52	23.40
			Test-retest (*n* = 37)	21	56.80
Type of sport		Individual sport	Total (*N* = 516)	138	26.70
			EFA (*n* = 294)	69	23.50
			CFA (*n* = 222)	69	31.10
			Test-retest (*n* = 37)	18	48.60
		Team sport	Total (*N* = 516)	378	73.30
			EFA (*n* = 294)	225	76.50
			CFA (*n* = 222)	153	68.90
			Test-retest (*n* = 37)	19	51.40
Governorates	Total *(N* = 516)	Tunis		114	22.10
		Sfax		102	19.80
		Kairouan		101	19.60
		Gafsa		110	21.30
		Gabes		89	17.20

*Note*. EFA: exploratory factor analysis; CFA: confirmatory factor analysis.

### Measurement

The Basic Needs Satisfaction in Sport Scale (BNSSS) consists of twenty items that measure five factors of basic needs in sport: five items for each of the two dimensions (competence (COMP) and relatedness (RELAT)) and 10 items for the three forms of autonomy (four items for autonomy-choice (Auto.choice), three items for autonomy-volition (Auto.volition), and three items for autonomy-internal perceived locus of causality (Auto.IPLOC). The BNSSS was created by Ng, Lonsdale [20]. This instrument’s items use Likert scales ranging from 1 (Not true at all) to 7 (Very true). The highest numerical level corresponds the highest level of satisfaction, with the exception of the item five: “In my sport, I feel that I am being forced to do things that I don’t want to do” (belongs to autonomy-volition) which was formulated inversely (i.e., the highest numerical index corresponds the lowest value of satisfaction).

### Procedure

We utilized a translation and back-translation procedure to obtain the adaptation of the Arabic version of the BNSSS-20. This trans-cultural validation respected the International Test Commission (ITC) guidelines [38, 39] for adapting and translating tests. The translation of this scale was carried out by two bilingual translation teams characterized by their in-depth knowledge of the target language and the source language: first, a pair of two translators independently translated the original version into Arabic. The two versions were combined into a single version after a thorough check between them. Then, another team of two translators translated the two versions from Arabic to English in the same way without any reference to the original version. Finally, the completed version was compared with the original scale.

The article "Preliminary validity of the BNSSS-20 in Arabic: Exploratory study on basic needs satisfaction in sport for a sample of Tunisian athletes" was retracted in 2025. Reasons: unreliable data; unreliable results or conclusions; lack of ethics approval or compliance; missing or withdrawn patient consent.

We explained to the club coordinators the objectives of the study. The instruments were distributed to the teams before the training session. The BNSSS-20 was typically completed two hours before the start of athletic competitions. The instructions of the scale were well described to the athletes. The athletes also reported their age, gender and sport discipline.

The study was fully approved by the ethics committee of the National Center of Medicine and Sciences in Sport of Tunisia (approval number LR09SEP01) before the commencement of the assessments. For non-adult athletes, we asked for their parents’ permission. Verbal informed consent was obtained from each athlete before starting the study. The participation of the athletes was voluntary. The raw values collected by the athletes were processed to ensure maximum confidentiality.

### Statistical analysis

Data were processed using the software programs JASP (Version 0.16.3.0), the "Statistical Package for Social Sciences" SPSS (Version 24, IBM, Armonk, NY, USA) and AMOS (Version 24, IBM, Armonk, NY, USA).

First, the data were normally distributed in terms of skewness (Sk) and kurtosis (Kr) (see Table 1). Values between +2 and -2 are designated acceptable for a normal distribution [40, 41].

Multiple aspects of reliability were tested. Stability was determined by the level of correlation between the athletes’ responses [42]. The reliability of the BNSSS-20 was calculated by test-retest reliability (Bivariate correlations, Intra-Class Correlation) (See Table 3 The internal reliability of the instrument BNSSS-20 was tested by Cronbach’s α, McDonald’s ω, and Gutmann’s λ6 [43–45]. Internal consistency indicates the degree of inter-correlation between items on the BNSSS-20 [46]. The recommended reliability threshold for these indices is set at 0.70 for acceptability and 0.80 for good reliability.

Before EFA, is necessary to verify adequate sample size. The applied criterion for an adequate sample size for EFA is a subjects-to-variables ratio of 4:1 or 5:1 [47, 48]. Our study population was 14 times larger than the number of items (294 athletes vs. 20 items), which is determined to be "good" [49]. Second, to determine the factor structure of the instrument, an orthogonal Varimax-type exploratory factor analysis (EFA) according to Kaiser’s [50] Varimax criterion with a principal-component analysis (PCA) was applied to our scale from the 20 items of the survey [51]. No items were retained if they had a factor loading of 0.40 or less [52, 53]. The adequacy of this sample was measured by the Kaiser-Meyer-Olkin (KMO) statistic [54, 55].

The article "Preliminary validity of the BNSSS-20 in Arabic: Exploratory study on basic needs satisfaction in sport for a sample of Tunisian athletes" was retracted in 2025. Reasons: unreliable data; unreliable results or conclusions; lack of ethics approval or compliance; missing or withdrawn patient consent.

Finally, we used the widely recommended criterion for sample size measure for confirmatory factor analysis (CFA), which is sample size of participants to number of parameters ratio with a minimum of 5:1 and a maximum of 10:1 [56]. Our sample size passed the maximum requirement of 200 (222 athletes vs. 20 items). A confirmatory factor analysis (CFA) of the first order with maximum likelihood estimation was tested the factor structure in five dimensions of BNSSS-20. The analyses included various indices measuring the fit of the evaluated model. To test the fit of the models, the following indices were emphasized: the Goodness of Fit Index (GFI) [57], and the Adjusted goodness of fit index (AGFI), which must be equal to or higher than 0.85 and 0.90, respectively [58], the Comparative Fit Index (CFI) is a normed fit index between 0 and 1, the most accepted measure of good fit is a CFI ≥ 0.95 [59], the Not Normed Fit Index (NNFI) is based on the Tucker-Lewis Index, which was created through factor analysis, an index value of 0.9 or above indicated a good or excellent fit for both fit indices [60], Hu and Bentler [61] suggest that a good fit for the Standardized Root Mean Square Residual (SRMR) is less than 0.08, the Parsimony Normed Fit Index (PNFI), and the Parsimony Comparative Fit Index (PCFI) greater than 0.5 [62], for the Root Mean Square Error of Approximation (RMSEA), MacCallum, Browne [63] selected 0.01, 0.05, and 0.08 to indicate excellent, good, and mediocre fit respectively, and commonly applied χ ^2^ statistic (χ ^2^/ df ratio of 3 or less). The model fit of the retained data depends on a non-significant value of χ ^2^ [64]. Furthermore, an analysis of sensitivity (variance analysis, ANOVA) was performed to identify the effect of age, gender, and kind of sport on the scores of each factor of the instrument.

## Results

### Instrument quality

The basic characteristics of the sample population are present in **Table 1.**

**Table 2** examines the descriptive characteristics of the 20-item BNSSS. The means, standard deviations, kurtosis, and skewness of the dimensions are reported in this table.

**Table 2:** Descriptive statistics and normality of the 20-Item BNSSS (*N* = 294).

Item	M	SD	Sk	Kr (Zero Centered)
1	5.59	1.132	-1.023	1.292
2	4.21	1.978	-0.248	-1.216
3	5.16	1.496	-0.841	0.305
4	5.44	1.353	-1.011	0.655
5	5.17	1.503	-0.821	0.342
6	5.05	1.632	-0.851	-0.010
7	5.63	1.055	-1.099	1.384
8	5.14	1.479	-0.828	0.110
9	5.56	1.280	-1.198	1.363
10	5.62	1.187	-0.935	1.021
11	5.10	1.643	-0.864	0.081
12	5.06	1.662	-0.893	0.015
13	5.45	1.349	-1.067	0.846
14	4.97	1.648	-0.733	-0.219
15	4.15	1.904	-0.157	-1.153
16	4.10	2.010	-0.197	-1.298
17	5.05	1.583	-0.802	-0.208
18	5.56	1.106	-0.950	1.454
19	5.54	1.179	-0.760	0.429
20	5.55	1.318	-1.038	0.855

*Note*. M: Mean; SD: Standard deviation; Sk: Skewness; Kr: Kurtosis.

The article "Preliminary validity of the BNSSS-20 in Arabic: Exploratory study on basic needs satisfaction in sport for a sample of Tunisian athletes" was retracted in 2025. Reasons: unreliable data; unreliable results or conclusions; lack of ethics approval or compliance; missing or withdrawn patient consent.

Furthermore, the mean and standard deviation of the BNSSS-20 subscales by age are shown in **Table 3**.

**Table 3:** Distribution of the BNSSS-20 subscales by age (*N* = 294).

Age		COMP	Auto.choice	Auto.volition	Auto.IPLOC	RELAT
[14–18]	M	24.86	21.29	15.09	11.23	27.65
	SD	7.25	5.36	4.49	5.87	5.61
[19–28]	M	25.82	23.16	16.09	14.44	28.43
	SD	8.28	3.95	3.80	4.49	4.12

*Note*. M: Mean; SD: Standard deviation; COMP: competence; Auto.choice: autonomy-choice; Auto.volition: autonomy-volition; Auto.IPLOC: autonomy-internal perceived locus of causality; RELAT: relatedness.

The stability over time for the BNSSS-20 was analyzed using the test-retest consistency index. 37 athletes (16 males, 21 females; mean age 19.51 ± 3.95 years; 14 to 25) responded to the measurement scale. After four weeks, the same group completed the same instrument. The test-retest sample is part of the overall study population. This was a homogeneous population regarding age and gender. The temporal stability (test-retest reliability) of the BNSSS-20 was verified by correlational analysis between BNSSS-20 scores collected by 37 individuals on two occasions four weeks apart. The correlation coefficient was .799 (*p* < 0.001), designating good temporal stability of the instrument. However, the bivariate correlation coefficient does not account for systematic differences, and some authors have suggested using the intraclass coefficient (ICC) as a standard parameter for absolute agreement instead of the correlation coefficient [65]. A minimum sample size of 22 participants is required to detect an ICC value of 0.50 for 80% power with alpha fixed at 0.05 [66]. In case of possible dropout in the retest phase, an additional twenty percent of the minimum sample is suggested, resulting in a target number of 27 participants. Hence, the number of 37 participants in this work was sufficient to determine the instrument’s temporal stability. Therefore, the intraclass coefficient (ICC) was 0.847, indicating excellent temporal stability of the tool (see **Table 4** and **Fig 1**).

**Fig 1:** The relationship between the BNSSS-20 scores reported at time 1 and time 2.

The article "Preliminary validity of the BNSSS-20 in Arabic: Exploratory study on basic needs satisfaction in sport for a sample of Tunisian athletes" was retracted in 2025. Reasons: unreliable data; unreliable results or conclusions; lack of ethics approval or compliance; missing or withdrawn patient consent.

**Table 4:** Test-retest reliability of the BNSSS-20 (*n* = 37).

	Test-retest reliability	
	Bivariate correlations	Intra-class correlation
BNSSS	0.79***	0.84
IC 95%	0.64–0.89	0.55–0.93

*Note*.

*** Statistically significant at *p* < 0.001.

As indicated in **Table 5**, the internal consistency of the Arabic version BNSSS-20 was good.

**Table 5:** Internal consistency of the Arabic version of the BNSSS-20 (*N* = 294).

Scale	Cronbach alpha (CI 95%)	McDonald’s omega (CI 95%)	Gutmann’s λ6 (CI 95%)
BNSSS (Normal-Scaled Items)	0.886 (0.865–0. 905)	0.773 (0.736–0.810)	0.970 (0.965–0.977)
BNSSS (Reverse-Scaled Items)	0.849 (0.822–0.872)	0.754 (0.715–0.794)	0.964 (0.958–0.973)

*Note*. The following item correlated negatively with the scale: Item 5.

We examined the inter-item correlation coefficients to quantitatively measure the internal consistency of the BNSSS scale [67]. **Table 6** provides a matrix of correlation coefficients. Generally, all items are positively and moderately correlated with each other. Some exceptions occurred between the correlations of item 2 and item 1, and item 2 and item 10, where there was no apparent correlation. Item 2 refers to autonomy-volition. Autonomy appears to be the most important factor, due to its high association with intrinsic motivation [68]. A social context that enhances the feeling of need for autonomy allows for choices to be selected and initiative to be taken [11]. According to Reeve, Nix [19], autonomy-volition refers to a choice of action without pressure. Therefore, the experience should be characterized by great flexibility and light pressure during action. In addition, coaches who foster a performance climate have a negative impact on athletes’ basic needs and motivation [69]. Instead of simply offering imposed directives, athletes may also need to feel free and initiative in their action in order to promote optimal motivation and maximum performance towards their sport.

**Table 6:** Inter-item correlation matrix coefficients for the 20-Item BNSSS (*N* = 294).

	1	2	3	4	5	6	7	8	9	10	11	12	13	14	15	16	17	18	19	20
1	1.000																			
2	-0.018	1.000																		
3	0.080	0.362	1.000																	
4	0.384	0.025	0.157	1.000																
5	0.120	0.384	0.862	0.148	1.000															
6	0.146	0.115	0.286	0.171	0.264	1.000														
7	0.786	0.099	0.060	0.354	0.093	0.162	1.000													
8	0.141	0.411	0.845	0.150	0.871	0.278	0.116	1.000												
9	0.373	0.099	0.228	0.873	0.207	0.150	0.327	0.218	1.000											
10	0.752	-0.001	0.058	0.453	0.086	0 .184	0.750	0.084	0.438	1.000										
11	0.124	0.164	0.260	0.176	0.317	0.909	0.189	0.294	0.153	0.190	1.000									
12	0.186	0.137	0.306	0.164	0.320	0.862	0.215	0.348	0.147	0.209	0.863	1.000								
13	0.363	0.077	0.173	0.814	0.171	0.120	0.326	0.196	0.797	0.414	0.139	0.109	1.000							
14	0.157	0.183	0.250	0.137	0.273	0.879	0.191	0.275	0.127	0.192	0.878	0.862	0.104	1.000						
15	0.033	0.928	0.356	0.052	0.381	0.103	0.147	0.405	0.120	0.040	0.134	0.114	0.086	0.156	1.000					
16	0.034	0.838	0.369	0.001	0.361	0.145	0.102	0.373	0.089	0.039	0.149	0.173	0.063	0.196	0.806	1.000				
17	0.153	0.148	0.311	0.192	0.305	0.817	0.138	0.302	0.161	0.159	0.796	0.785	0.115	0.846	0.111	0.175	1.000			
18	0.774	0.043	0.053	0.385	0.102	0.164	0.778	0.119	0.378	0.740	0.147	0.187	0.343	0.194	0.074	0.102	0.178	1.000		
19	0.773	0.000	0.052	0.331	0.091	0.181	0.800	0.103	0.314	0.756	0.164	0.213	0.296	0.201	0.038	0.037	0.168	0.776	1.000	
20	0.354	0.042	0.203	0.852	0.195	0.109	0.365	0.205	0.839	0.414	0.110	0.090	0.811	0.078	0.051	0.021	0.101	0.391	0.329	1.000

The article "Preliminary validity of the BNSSS-20 in Arabic: Exploratory study on basic needs satisfaction in sport for a sample of Tunisian athletes" was retracted in 2025. Reasons: unreliable data; unreliable results or conclusions; lack of ethics approval or compliance; missing or withdrawn patient consent.

### Exploratory factor analysis

The KMO statistic indicated a good sampling adequacy (KMO = 0.868, Bartlett’s test of sphericity *p* < 0.001) and included five independent principal factors whose eigenvalues were above the threshold indicated by Cattell [70] and Kaiser [71]. The five factors together explained 87.30% of the variance in the data. The eigenvalue of the first principal component of competency (COPM) explained 33.49% of the total variance (eigenvalue = 6.69), while the second principal component of membership (RELAT) accounted for 20.80% of the total variance (eigenvalue = 4.16), 14.94% (eigenvalue = 2.98), 10.75% (eigenvalue = 2.15), and 7.30% (eigenvalue = 1.46). The factor loadings of the items from the EFA for the five-factor model were between 0.836 and 0.948 (reported in **Table 7**). Only values above 1 were retained.

**Table 7:** Factor structure of the BNSSS-20 in the Arabic language (*N* = 294).

Items in Arabic language	Components				
	1	2	3	4	5
يمكنني التغلب على التحديات في رياضتي	0.943				
أنا ماهر في رياضتي	0.936				
أشعر أنني جيد في رياضتي	0.909				
لدَيَّ فرص لأشعر أنني جيد في رياضتي	0.940				
لدَيَّ القدرة على الأداء الجيد في رياضتي	0.885				
في رياضتي، لدَيَّ فرص لاتخاذ الخيارات			0.916		
في رياضتي، لدَيَّ رأي في كيفية سير الأمور			0.905		
في رياضتي، يمكنني المشاركة في عملية اتخاذ القرار			0.888		
في رياضتي، أحصل على فرص لاتخاذ القرارات			0.902		
أشعر أنني أشارك في رياضتي عن طيب خاطر					0.907
في رياضتي، أشعر أنني مجبر على فعل أشياء لا أريد القيام بها					0.912
أختار ممارسة رياضتي بمحض إرادتي					0.898
في رياضتي، أشعر أنني أسعى لتحقيق أهدافي الخاصة				0.948	
في رياضتي، لدي شعور بالرغبة في أن أكون هناك				0.938	
في رياضتي، أشعر أنني أفعل ما أريد أن أفعله				0.899	
في رياضتي، أشعر أنني قريب من الآخرين		0.884			
أبدي اهتماما بالآخرين في رياضتي		0.894			
هناك أشخاص في رياضتي يهتمون بي		0.836			
في رياضتي، هناك أشخاص يمكنني الوثوق بهم		0.875			
لدَيَّ علاقات وثِقة بالآخرين في رياضتي		0.900			

(English translation of the items). Item 1. I can overcome challenges in my sport. Item 2. I am skilled at my sport. Item 3. I feel I am good at my sport. Item 4. I have opportunities to feel that I am good at my sport. Item 5. I have the ability to perform well in my sport. Item 6. In my sport, I have opportunities to make choices. Item 7. In my sport, I have a say in how things are done. Item 8. In my sport, I can participate in the decision-making process. Item 9. In my sport, I get opportunities to make decisions. Item 10. I feel like I am participating in my sport willingly. Item 11. In my sport, I feel that I am being forced to do things that I don’t want to do. Item 12. I choose to practice my sport of my own free will. Item 13. In my sport, I feel that I am pursuing my own goals. Item 14. In my sport, I really have a sense of wanting to be there. Item 15. In my sport, I feel I’m doing what I want to be doing. Item 16. In my sport, I feel close to the others. Item 17. I show concern for other people in my sport. Item 18. There are people in my sport who do care about me. Item 19. In my sport, there are people who I can trust. Item 20. I have relationships and trust with others in my sport.

The article "Preliminary validity of the BNSSS-20 in Arabic: Exploratory study on basic needs satisfaction in sport for a sample of Tunisian athletes" was retracted in 2025. Reasons: unreliable data; unreliable results or conclusions; lack of ethics approval or compliance; missing or withdrawn patient consent.

The internal consistency of the Arabic version of scale calculated by Cronbach’s alpha determined that it had good internal reliability (α BNSSS-20 = 0.886, 95% IC = 0.865–0.905) [72]. Also, the reliability of the instrument provided by Gutmann λ6 values was excellent (λ6 BNSSS-20 = 0.970, 95% CI = 0.965–0.977). Furthermore, the internal consistency measured by McDonald’s omega (ω BNSSS-20 = 0.773, 95% CI = 0.736–0.810) was satisfactory. McDonald’s omega is a better indicator of internal consistency for the instrument [73] (see **Table 3**).

### Confirmatory factor analysis

The CFA performed multiple model fit indices according to the criteria of several researchers. According to critical standards, the ideal standardized χ ^2^ (Chi-Square) value over the number of degrees of freedom (χ ^2^/df) should be placed between 2 and 3 (2 ≤ χ ^2^/df ≥ 3) Wheaton, Muthen [74] and Tabachnick and Fidell [75]. Consequently, for the Chi-Square and normalized χ ^2^ (χ ^2^/df) statistics, the collected indices were satisfactory for the model; see [76–78]. We calculated various fit indices (AGFI, GFI, CFI, NNFI (TLI), NFI, PNFI, PCFI, RMSEA, and SRMR), and the critical values for indices AGFI, GFI (see Tabachnick and Fidell [75]), NFI, CFI, and the NNFI (TLI) (see, Bryant and Yarnold [79], Hu and Bentler [59], Fan, Thompson [80], and Byrne [81]) must be greater than 0.95. However, the AGFI and GFI of the current scale were between 0.90 and 0.93; see, Schermelleh-Engel, Moosbrugger [58]. Some researchers consider the critical value above 0.90. PNFI and PCFI were greater than the adaptive value of 0.50 (PNFI = 0.81; PCFI = 0.83). Also, for RMSEA and SRMR, the value should not exceed 0.05; see Byrne [82]. In conclusion, the 20-item model showed for all tested indices an excellent fit to the theoretical model, justifying the factor structure for the Tunisian sport sample. The confirmatory factor analyses confirmed good fit for the five-factor Arabic version of BNSSS-20 model χ ^2^ = 184.585, degrees of freedom 160 at *p* < 0.08; CFI = 0.99; NFI = 0.96; CFI = NNFI (TLI) = IFI = 0.99; GFI = 0.93; AGFI = 0.91; SRMR = 0.02, and RMSEA = 0.02 (CI 90% = 0.02–0.04). Thus, the hypothesized parameters of this model were significant at *p* < 0.05 (**Table 8** and **Fig 2**).

The article "Preliminary validity of the BNSSS-20 in Arabic: Exploratory study on basic needs satisfaction in sport for a sample of Tunisian athletes" was retracted in 2025. Reasons: unreliable data; unreliable results or conclusions; lack of ethics approval or compliance; missing or withdrawn patient consent.

**Fig 2:** Standardized results of the confirmatory factor analysis (CFA) of the Arabic version of BNSSS (*N* = 222).

**Table 8:** Summary of fit indices for the BNSSS-20 confirmatory factor analysis models (*N* = 222).

Model	X^2^/df	AGFI	GFI	NFI	IFI = TLI = CFI	PNFI	PCFI	RMSEA (CI 95%)	SRMR
BNSSS	1.154	0.91	0.93	0.96	0.99	0.81	0.83	0.02 (0.01–0.04)	0.02

*Note*. χ^2^/df, relative chi-square; AGFI, Adjusted Goodness of Fit Index; GFI, Goodness of Fit Index; NFI, Normed Fit Index; IFI, Incremental Fil Index; TLI, Tucker Lewis Index; CFI, Comparative Fit Index; PNFI, Parsimony Normed Fit Index; PCFI, Parsimony Comparative Fit Index; SRMR, Standardized Root Mean Square Residual; RMSEA, Root Mean Square Error of Approximation.

### Sensitivity analysis

As determined by ANOVA, there was an effect of age on autonomy-internal perceived locus of causality. There was also an effect of sport type on autonomy-internal perceived locus of causality and autonomy-volition. The sensitivity analysis determined that athletes 19–28 years of age used all dimensions of basic need satisfaction in sport more than the participants of younger age (14–18 years). In the interaction effects, no significant influence could be identified (indicated in **Table 9**).

**Table 9:** Impact of age, sex, sport type (i.e., individual versus team sports), and their interaction effects on the dimensions of the basic needs’ satisfaction in sport BNSSS-20 (*N* = 294).

Variables	F				
	COMP	Auto.choice	Auto.volition	Auto.IPLOC	RELAT
Age	0.137	2.984	0.312	8.936**	1.793
Gender	3.080	3.111	0.311	0.146	1.795
Sport	3.339	0.464	9.871**	4.676*	0.006
Age X Gender	0.841	0.429	0.020	0.945	0.405
Age X Sport	0.195	0.493	2.238	1.800	1.126
Gender X Sport	0.856	1.641	1.301	0.214	1.833
Age X Sport X Gender	0.652	1.136	0.037	0.170	0.034

*Note*. COMP: competence; Auto.choice: autonomy-choice; Auto.volition: autonomy-volition; Auto.IPLOC: autonomy-internal perceived locus of causality; RELAT: relatedness

* Statistically significant at *p* < 0.05

** Statistically significant at *p* < 0.01.

The article "Preliminary validity of the BNSSS-20 in Arabic: Exploratory study on basic needs satisfaction in sport for a sample of Tunisian athletes" was retracted in 2025. Reasons: unreliable data; unreliable results or conclusions; lack of ethics approval or compliance; missing or withdrawn patient consent.

## Discussion

Our results suggested that the Arabic version of the BNSSS is a valid and reliable scale for assessing the level of satisfaction of basic needs in sport for athletes from different sport type (whether individual or collective) and both sexes. Overall, we found very good psychometric properties for this adapted scale. Moreover, the results obtained by the EFA suggested that this SBNNN-20 scale well reflected the expected theoretical model, with good internal consistency for all the adopted factors. The 20 BNSSS items showed excellent reliability (McDonald’s omega = 0.773, Cronbach’s α = 0.886, Gutmann’s λ6 = 0.970) and good temporal stability (ICC = 0.847). Similarly, the CFA fit indices were perfect (CFI = 0.99; NFI = 0.96; CFI = NNFI (TLI) = IFI = 0.99; GFI = 0.93; AGFI = 0.91, and SRMR = RMSEA = 0.02).

The internal reliability (test-retest) is adequate for the scale (*r* = 0.79 at *p* < 0.001) designating acceptable repeatability. Thus, good correlation resulted in adequate stability of the instrument over time. The obtained data of reliability over time (test-retest) are verified by the correlations between the BNSSS dimension values. Intra-class Correlation Coefficients (ICC) with 95% confidence intervals were determined to check the absolute agreement between the two times. The BNSSS-20 was stable over time over a 4-week period. Therefore, the sample size of 37 was suitable for measuring the temporal stability of the instrument. The absolute agreement between scores at both times with ICC with 95% confidence intervals and a 2-way random effects model was assessed by a mean score (k = 2) of BNSSS-20 [83]. The internal consistency of the scale calculated by Cronbach’s α, McDonald’s ω, and Gutmann’s λ6, was excellent. Thus, all values demonstrate good fidelity for the scale. To conclude, most dimensions constituted significant correlations with excellent values of the inter-item correlation coefficients.

In addition, the results of the EFA showed that this scale well reproduced the expected theoretical model (concerning homogeneity of the items) with an interesting internal consistency for all the extracted factors. Furthermore, the results of the CFA indicated a good fit to the theoretical model, validating in a satisfactory way the five-dimensional factor structure in a population of Tunisian athletes.

The article "Preliminary validity of the BNSSS-20 in Arabic: Exploratory study on basic needs satisfaction in sport for a sample of Tunisian athletes" was retracted in 2025. Reasons: unreliable data; unreliable results or conclusions; lack of ethics approval or compliance; missing or withdrawn patient consent.

In terms of methodology, item 11 was negatively correlated with the BNSSS-20 scale, which has a low factor load. This item is the only sentence in the opposite direction (“In my sport, I feel that I am being forced to do things that I don’t want to do”), which might explain this finding. Therefore, the internal consistency of the instrument will decrease with reverse-scaled items: α BNSSS-20 = 0.849 (IC 90%; 0.822–0.872), ω BNSSS-20 = 0.754 (IC 90%; 0.715–0.794), and λ6 BNSSS-20 = 0. 964 (IC 90%; 0.958–0.973). In contrast, the unfiltered internal consistency of item 5 is higher: α BNSSS-20 = 0.886, 95% CI = 0.865–0. 905, ω BNSSS-20 = 0.773, 95% CI = 0.736–0.810, and λ6 BNSSS-20 = 0.970, 95% CI = 0.965–0.977.

Finally, the results of the present study verify that there is a Tunisian version of the BNSSS with good psychometric properties, maintaining the five-dimensional factor structure suggested by Ng, Lonsdale [20] to assess the level of satisfaction of basic needs in sport in Tunisia, which is a step forward for sport psychology in creating a measurement instrument for all kinds of sports.

### Limitations

This study has some limitations. It is necessary to evaluate this measurement tool with more heterogeneous populations in additional Arabic-speaking countries in order to determine the general extensibility of the results and to examine the social factors affecting the satisfaction of basic needs in sports. Also, this sample was restrained to a cohort of very young athletes. Athletes after age 30 have different motivations, and it appears that motivations for engagement in sport may change throughout the lifespan [84]. likewise, basic needs persist over throughout lifetime, although their relative interest, and the ways in which they are met vary the lifespan and across cultures [6].

There is a need to develop tools related to the assessment of psychological needs in sport contexts. Basic needs affect the motivation and performance of athletes in sport development [68]. In the Arab world, studies that focus on basic needs in the context of sport remain rare. It is advisable to use this instrument to learn about the importance of meeting the needs of athletes from different cultural backgrounds and skill to various degrees.

## Conclusion

Finally, we can conclude that our study attempted to adjust the factor structure, internal reliability, validity, and sensitivity of the BNSSS-20. These results convincingly demonstrate satisfactory stability over time (test-retest), very good internal reliability, good correlation values, good EFA factor structure and excellent CFA fit indices. Furthermore, the sensitivity analysis revealed the effect of two variables (i.e., age, sport type) on some factor scores of basic needs in sport. In conclusion, this adapted instrument is a good tool to quantitatively assess the level of satisfaction of basic needs in sport (whether individual or collective) for athletes in Arabic-speaking countries.

The article "Preliminary validity of the BNSSS-20 in Arabic: Exploratory study on basic needs satisfaction in sport for a sample of Tunisian athletes" was retracted in 2025. Reasons: unreliable data; unreliable results or conclusions; lack of ethics approval or compliance; missing or withdrawn patient consent.

## Supporting information

S1 Data (XLSX)

S2 Data (XLSX)

S3 Data (XLSX)

S4 Data (XLSX)

S1 File Arabic version and original version of BNSSS-20. (DOCX)
